# Malalignment and distal contact of short tapered stems could be associated with postoperative thigh pain in primary total hip arthroplasty

**DOI:** 10.1186/s13018-021-02215-w

**Published:** 2021-01-19

**Authors:** Zhijie Chen, Bin Li, Kaizhe Chen, Jianmin Feng, Yi Wang, Zhihong Liu, Chuan He

**Affiliations:** Department of Orthopaedics, Shanghai Key Laboratory for Prevention and Treatment of Bone and Joint Diseases, Shanghai Institute of Traumatology and Orthopaedics, Ruijin Hospital, Shanghai Jiao Tong University School of Medicine, 197 Ruijin 2nd Road, Shanghai, 200025 People’s Republic of China

**Keywords:** Distal contact, Stem malalignment, Short tapered stem, Thigh pain, Total hip arthroplasty

## Abstract

**Purpose:**

Short tapered stem placement has been extensively employed in total hip arthroplasty (THA). Suboptimal fixation tends to cause postoperative complications, such as thigh pain. However, it remains unclear whether poor seating/alignment of short tapered stems contributes to thigh pain. In this study, we retrospectively examined the factors that might be associated with thigh pain.

**Methods:**

Medical records of 230 patients who had undergone THAs at our hospital were reviewed retrospectively. All patients received the same mediolateral (ML) short tapered femoral stems. The association between thigh pain and patients’ demographics, radiographic findings, or the type of fitting of the femoral stems was investigated.

**Results:**

In our cohort, 68 patients (27.8%) presented with thigh pain. Among 203 type I fit patients, 62 (30.5%) developed thigh pain, while only 6 out of 43 (12.2%) type II fit patients had thigh pain, with the differences being statistically significant (*x*^2^ = 6.706, *p* = 0.01). In addition, hip anteroposterior radiographs exhibited that the stem angulation (mean 2.52°), the variation in angulation (mean 1.32°), and the extent of femoral stem subsidence (mean 0.29 cm) were greater in patients with thigh pain than in their counterparts without thigh pain (all *p* < 0.05).

**Conclusion:**

Malalignment and improper seating of short tapered stems could be at least one of the reasons for post-THA thigh pain. The distal contact between the stem tip and the medial femoral cortex might result in thigh pain. Our study suggested that distal implant contact should be avoided, and stem alignment should be meticulously performed in the placement of ML short tapered femoral stems for THA.

## Introduction

Total hip arthroplasty (THA) represents one of the most successful and cost-effective operations of modern medicine [1]. In spite of this, researchers are still endeavoring to improve the mechanical and biological properties of hip prostheses. Cementless femoral fixator with tapered-geometry designs has evolved substantially over the past several decades, and the research effort is now being directed at shorter stems. As a result, short tapered stems have been increasingly used in THA over the past decade. The stems are characterized by reduced neck geometry, intuitive sizing, and curved distal tip, thereby rendering surgery less invasive and recovery quicker since incisions are smaller [2, 3]. Furthermore, they only require more straightforward femoral preparation with a “broach-only” system without distal reaming, and their bone-conserving nature can create a more favorable condition at the potential revision site [4–6].

Although short tapered stems were reportedly performed as well as standard ones, with equally good functional improvement, pain relief, and implant survival, mounting evidence still shows that thigh pain remains a common complication after THA [3, 7, 8]. For instance, a 2- to 4-year follow-up by Amendola et al. revealed that, after THA with a short tapered stem, 16% of the patients (226 in all) developed mild thigh pain and 9% suffered from moderate or severe thigh pain [3]. The pain has been considered to be of intermittent and self-limiting nature and does not necessitate medication [9–11], and it has not been deemed as a serious problem by most surgeons. Persistent thigh pain after THA typically develops around 2 years after operation [12], and it is both patient- and implant-related. Mechanistically, thigh pain seems to be multifactorial, involving the design, size, elastic modulus, extent of porous coating of the stem, and architecture of the proximal femur [13, 14].

So far, no consensus has been reached regarding the optimal seating of short tapered stems in the femoral metaphysis. Compared to conventional stems, it is more difficult to ensure appropriate alignment and seating of short tapered stems. Apart from implant/bone contact at the metaphysis, to ensure stability, the distal contact between the stem tip and the medial femoral cortex is required in most cases. The operation, in turn, might lead to misalignment of the stem to some extent. Unfortunately, it remains unclear whether poor seating/alignment of short tapered stems causes thigh pain. In this study, we retrospectively investigated the factors that might be associated with thigh pain after THA with short tapered stem.

## Materials and methods

Upon approval by the institutional review board of our hospital, we performed a retrospective analysis of relevant data from our electronic medical record system. Included in the analysis were 289 patients (322 hips) who had undergone primary THA from October 2015 to August 2018. Of them, 230 patients (involving 252 hips) had complete follow-up data. The stem used in this study was titanium, circumferentially and proximally coated mediolateral (ML) taper short femoral stem (Tri-Lock BPS, DePuy Synthes, Johnson and Johnson, Warsaw, IN), and was implanted with a 32- or 36-mm modular ceramic femoral head (BIOLOX Delta). The stem length (95–119 mm) increased with ML size. The acetabular component was implanted with the Pinnacle acetabular component (DePuy Synthes, Johnson and Johnson, Warsaw, IN) in all hips. Ceramic liners (BIOLOX Delta) were used in all hips.

The inclusion criteria for this case series study were patients who had undergone THA due to osteoarthritis, acute fracture (displaced femoral neck fractures), developmental dysplasia (Crowe I or II), aseptic necrosis, avascular necrosis, drug-induced necrosis, and post-traumatic arthritis, among others. The exclusion criteria were patients who were diagnosed as having hemophilic arthritis and had undergone intramedullary nailing or total knee arthroplasty. Patients with any comorbidities causing thigh pain before the THA were not included.

All procedures were performed by three surgeons via a direct anterior (32 hips), anterior-lateral (142 hips), or minimal invasive posterolateral approach (78 hips). The stem was inserted with a broach-only technique, and a similar broaching technique was used across the 3 surgeons. For all cases, the acetabulum was reamed to 1 mm less than the diameter of the component used. Dome screws were used to augment fixation at the surgeon’s discretion. Patients were allowed to progress to full weight bearing as tolerated, typically transitioning from a walker or crutches to a cane to no support over a period of 4 weeks.

Among the selected cases, the mean age of the patients at the time of the primary THA was 61 years (range 23–84 years), and there were 72 men and 158 women. Clinical follow-up lasted for a mean time of 2.7 years (range, 1.5–4.6 years). Follow-up evaluation covered the Harris Hip Score (HHS) [15], history and examination, and determination of whether future revision surgery was planned. The HHS was obtained before operation (acute fractures not included) and at every follow-up visit. Postoperative complaints, such as thigh pain, were recorded at each visit. Whether the pain occurred at rest or during activity was not specified. If a patient demanded an explanation of “thigh pain,” she or he was told that it was pain below the hip but above the knee. If a patient reported such pain, she or he was asked whether pain was intermittent or persistent and when it had commenced [16, 17]. The hips were divided into two groups (thigh pain group and no thigh pain group; patients who had undergone bilateral THAs could have pain in one or both hips).

Radiographs were taken within 3 days before surgery and 1 day, 6 weeks, 3, 6 months, 1 year after surgery, and then on annual basis. Patients returned to the clinic for follow-up. If they were unable to return, radiographs were taken elsewhere and were sent to us for evaluation. The radiographs included anteroposterior (AP) views of the pelvis that involved the tip of the femoral prosthesis and AP and lateral views of the femur that included the hip.

All preoperative and postoperative radiographs were retrospectively analyzed, and radiological parameters were measured and checked by two authors. The following parameters were collected (Figs. 1 and 2):

1. Preoperative AP radiographs of the hip (Fig. 1a): (*d*) metaphyseal diameter 2 cm above the level of the lesser trochanter midpoint, (*e*) isthmus diameter which represents the width of the narrowest part of the proximal femoral canal, (*f*) diameter of the femoral shaft which was measured 10 cm distal to the center of the small trochanter, and (*g*) internal width of the medullar canal which was measured 10 cm distal to the center of the small trochanter. Femoral flare index (FFI) was obtained through the ratio between the metaphyseal diameter 2 cm above the level of the lesser trochanter midpoint (*d*) and isthmus diameter (*e*). Femoral cortical index (FCI) was obtained through the ratio between the thickness of cortical bone (*f*, *g*) and the diameter of the femoral shaft (*f*) measured 10 cm distal to the center of the small trochanter.
2. Postoperative AP radiographs of the hip (Figs. 1and 2b ,a, c): (*h*) the width of the stem which was measured at the proximal end of stem tip arc; (*i*) the internal width of medullar canal, which was measured at the proximal end of tip arc; (*j*) the width of the stem, which was measured at the distal end of porous coating; (*k*) the internal width of medullar canal, which was measured at the distal end of porous coating; (*α*_1_) coronal stem angulation (CSA), which represents the angle between the stem axis and the femur axis at the first follow-up; (*α*_2_) CSA, which is representative of the angle between the stem axis and the femur axis measured at the last follow-up; (*s*_1_) distance between the major trochanter apex and the stem shoulder perpendicular to the femoral stem axis measured at the first follow-up; and (*s*_2_) distance between the major trochanter apex and the stem shoulder perpendicular to the femoral stem axis at the last follow-up. Stem-intramedullary canal diameter ratio (S-ICDR) at the proximal end of the stem tip arc is the ratio between the diameter of stem (*h*) and the diameter of intramedullary canal (*i*) at the proximal end of the stem tip arc. S-ICDR at the distal end of porous coating is the ratio between the diameter of stem (*j*) and the diameter of intramedullary canal (*k*) at the distal end of porous coating. Femoral stem subsidence (FSS) from the first to last follow-up visits is the difference between the distance at the first follow-up (*s*_1_) and the distance at the last follow-up (*s*_2_). Variation in coronal stem angulation (VCSA) from the first to last follow-up visits was obtained by subtracting the stem angulation at the first follow-up (*α*_1_) from the stem angulation at the last follow-up (*α*_2_).
3. Postoperative lateral radiographs of the hip (Figs. 1, 2c and b): (*β*) sagittal stem angulation (SSA), which represents the angle between the stem axis and the femur axis at the first follow-up.

**Fig. 1:** **a**–**c** A representative image for type II fit. This patient was a 66-year-old woman who underwent THA at age 65 using a short tapered stem. **a** A preoperative AP radiograph of her left hip. **b** A 6-month postoperative AP radiograph of the hip. **c** A 6-month postoperative lateral radiograph of the hip. The following parameters were measured: (*d*) metaphyseal diameter 2 cm above the level of the lesser trochanter midpoint, (*e*) isthmus diameter which represents the width of the narrowest part of the proximal femoral canal, (*f*) diameter of the femoral shaft which is measured 10 cm distal to the center of the small trochanter, (*g*) internal width of the medullar canal which is measured 10 cm distal to the center of the small trochanter, (*h*) width of the stem which is measured at the proximal end of stem tip arc, (*i*) internal width of the medullar canal which is measured at the proximal end of the tip arc, (*j*) width of the stem which is measured at the distal end of porous coating, and (*k*) internal width of the medullar canal which is measured at the distal end of porous coating

**Fig. 2:** **a**–**c** A representative image for type I fit. This patient was a 62-year-old woman who underwent THA at age 60 using a short tapered stem, which is a type I fit. **a** A postoperative AP radiograph of her left hip. **b** A postoperative lateral radiograph of the hip. **C** A 6-month postoperative AP radiograph. The following parameters were measured: (*α*_1_) CSA, which represents the angle between the stem axis and the femur axis at the first follow-up; (*α*_2_) CSA, which represents the angle between the stem axis and the femur axis at the last follow-up; (*s*_1_) distance between the major trochanter apex and the stem shoulder perpendicular to the femoral stem axis at the first follow-up; (*s*_2_) distance between the major trochanter apex and the stem shoulder perpendicular to the femoral stem axis at the last follow-up; and (*β*) SSA, which represents the angle between the stem axis and femur axis at the first follow-up. In the AP radiograph, if *α*_1_/*α*_2_ > 0, it illustrates the stem alignment is valgus, and if *α*_1_/*α*_2_ < 0, it illustrates the stem alignment is varus. In the lateral radiograph, if *β* > 0, it illustrates the stem alignment is retroverted, and if *β* < 0, it illustrates the stem alignment is anteverted

Stem subsidence was diagnosed when a stem subsided more than 4 mm, as measured on a perpendicular line drawn from the greater trochanter to the lateral border of the implant. And implant loosening was diagnosed when a stem sunk more than 4 mm and/or varus/valgus migration range was greater than 5° [7]. Stem alignment is usually defined as neutral, valgus (lateral deviation> 5°), or varus (medial deviation> 5°) [18]. However, we did not use these values in favor of a more precise definition of stem alignment, which, we believe, is more helpful in clinical practice. The sagittal angle (on lateral radiographs) was defined as positive if the stem alignment was retroverted, and negative if it was anteverted. Similarly, the coronal angle (in AP radiographs) was deemed positive if the stem alignment was valgus, and negative if it was varus. Thus, “varus/valgus” merely reflects the extent of alignment deviation or the magnitude of stem angulation.

In previous studies, the implant fit was evaluated on the basis of the amount of implant/bone engagement as described by Faizan et al. [19]. In this study, we made some modifications to re-define the implant fit: the type I fit indicates a contact between the stem tip and the adjacent cortical bone, while there has no distal contact with type II fit. Logistic regression analysis was performed on baseline characteristics, such as implant fit, to further identify the risk factors of thigh pain.

Pearson chi-square was used for categorical variables, Student *t* tests for continuous variables, and logistic regression for risk factor analysis. All statistical analyses were conducted using SPSS version 20.0. A *p* value < 0.05 was considered statistically significant.

## Results

Of the 230 patients (252 hips) included in the study, 72 (31%) were male and 158 (69%) were female. Twenty-two patients underwent bilateral THAs, with a mean age of 61 ± 11 years at the surgery. The preoperative diagnoses included osteoarthritis in 82 (32.5%) hips, acute fracture in 54 (21.4%) hips, developmental dysplasia in 42 (16.7%) hips, aseptic necrosis in 33 (13.1%) hips, avascular necrosis in 25 (9.9%) hips, drug-induced necrosis in 11 (4.4%) hips, and post-traumatic arthritis in 5 (2.0%) hips. There existed no statistically significant differences in demographics or diagnoses between the two groups (Table 1).

**Table 1:** Characteristics of the patients between the pain group and the no-pain group

Characteristic	Thigh pain group	No thigh pain group	*p* value
Patients (number)	64	166	
Primary hips (number)	68	184	
Average age (years)	59.7 (29~84)	61.2 (23~84)	.345
Gender			.519
Male	18 (28.1%)	54 (32.5%)	
Female	46 (71.9%)	112 (67.5%)	
Preoperative diagnosis			.802
Osteoarthritis	23 (33.8%)	59 (32.1%)	
Acute fracture	16 (23.5%)	38 (20.7%)	
Developmental dysplasia	10 (14.7%)	32 (17.4%)	
Aseptic necrosis	9 (13.2%)	24 (13.0%)	
Avascular necrosis	8 (11.8%)	17 (9.2%)	
Drug-induced necrosis	2 (2.9%)	9 (4.9%)	
Post-traumatic arthritis	0	5 (2.7%)	
Implant fit			.010
Type I	62 (91.2%)	141 (76.6%)	
Type II	6 (8.8%)	43 (23.4%)	

The preoperative HHS was 44.8 (± 14), and at the last follow-up, the mean HHS was 89.2 (± 12), indicating that significant improvement was achieved (*p* < 0.01). There were 15 intra-operative calcar fractures, which were stabilized with one or two wires and were managed with the same recovery protocol. Two of 15 calcar fracture cases complained of temporary thigh pain. No femoral components were revised for aseptic loosening, periprosthetic joint infection, or prosthetic dislocation. Two patients had delayed wound healing. They were treated conservatively and recovered eventually.

In our cohort, 68 patients (27.8%) reported thigh pain after THA. As shown in Fig. 3, the reported thigh pain could be categorized into 3 groups: “not at first, but later” group (group 1), “persisted-for-some-time-and-then-vanished” group (group 2), and “all the time” group (group 3). Group 1 involved 10 hips (15%), group 2 had 36 hips (53%), and group 3 included 22 hips (32%). This finding indicated that thigh pain could develop at any time after THAs. What is more, 18% of the patients (45 hips) had mild thigh pain, 8% (20 hips) had moderate pain, and 1% (3 hips) had severe pain (Fig. 4).

**Fig. 3:** Postoperative thigh pain timeline. The report of thigh pain can be categorized into 3 groups: “not at first, but later” group, “persist for some time and then stop” group, and “all the time” group. Correspondingly, there were 15% (10 of 68) hips, 53% (36 of 68) hips, and 32% (22 of 68) hips for each group, respectively

**Fig. 4:** Patient-reported thigh pain from the visual analog scale. A total of 18% of patients (45 hips) had mild thigh pain, 8% (20 hips) had moderate, and 1% (3 hips) had severe thigh pain

Our main finding was that type I fits significantly higher in the thigh pain group than in the pain-free group. Among 68 patients with thigh pain, 62 (91.2%) were identified to be type I fit, while more type II fits were observed in the pain-free group (43 of 184, 23.4%), with the difference being statistically significant (*x*^2^ = 6.707, *p* = 0.01). The implant fit was associated with a clinically significant postoperative thigh pain (OR, 3.151; CI = 1.275~7.789; *p* = 0.013; Table 2).

**Table 2:** Logistic regression analysis of variables and thigh pain

Variable	Odds ratio	95% CI	*p* value
Implant fit	3.151	1.275 ~ 7.789	.013
Gender	0.002	–	.965
Age	1.509	–	.219
FFI	0.736	–	.391
FCI	0.389	–	.533
S-ICDR (e/f)	1.970	–	.160
S-ICDR (g/h)	3.644	–	.056

*FFI* femoral flare index, *FCI* femoral cortical index, *S-ICDR*, stem-intramedullary canal diameter ratio

In our study, no significant differences were found in FFI and FCI (*p* = 0.525 and *p* = 0.575), and femoral anatomical variation could not explain the thigh pain. Nonetheless, the mean CSA was 2.52° ± 1.84° and the mean SSA was 4.63° ± 1.83° in the pain group, while the CSA and SSA were 1.65° ± 1.42° and 3.96° ± 2.01°, respectively, in the pain-free group. We also found that the stem alignment was more valgus and retroverted in the pain group, since the CSA and SSA were more positive in this group than in the pain-free group (*p* = 0.001 and *p* = 0.016, respectively). In addition, there was a significant difference in VCSA scores between the pain and pain-free groups (1.32° ± 1.08° vs. 0.85° ± 0.93°, respectively, *p* = 0.004). Moreover, the FSS ranges averaged 0.29 cm ± 0.22 cm and 0.12 cm ± 0.12 cm in the pain and pain-free groups, respectively (*p* < 0.001). These significant differences suggest that the type I fit might be less stable than the type II fit. Collectively, our results indicated that the type I fit might bear an association with thigh pain.

## Discussion

With a mounting interest in less invasive surgery via smaller incisions, short tapered cementless stems have been increasingly used for femoral fixation. Clinically, though the functional and radiographic results were generally satisfactory, concern lingered since a significant portion of patients reported thigh pain. In this study, we examined 230 patients (252 hips involved) who had received ML short tapered femoral stems, with an attempt to understand the relationship between thigh pain and THA with short tapered stems. We compared the proximal and femoral anatomical structures (including the femoral flare and cortical indices), stem position relative to adjacent femoral cortical bone, and femoral stem fits in patients with and without thigh pain.

In our study, after the placement of short tapered stems, thigh pain developed in 27% (252 hips in all) of the patients about 1.5–4.6 years after surgery. Crawford et al. found that 15% (218 in all) of such patients reported anterior thigh pain and 15% complained of lateral thigh pain [20]. Richard et al. reported that 16% of patients (226 in all) had mild thigh pain and 9% suffered from moderate or severe thigh pain upon short taper stem replacement [21]. Our results were coincident with these previous findings. Although the incidence of thigh pain was relatively high, no patients had unbearable pain and had to undergo re-surgery. In another study by Cinotti et al., a more than 9-year follow-up revealed that 8% of patients (68 in all) reported thigh pain at the 2-year follow-up but only 3% did so at the last follow-up, and during this period, the pain was prosthesis-related [7]. This finding indicated some thigh pain might resolve naturally over time, and thigh pain could develop in any period of time after THA. The findings were consistent with the results of our study. Additionally, we found that, compared to pain-free patients, the CSA values were greater in patients with pain, and implant alignment was thus more varus/valgus in these patients. McCalden et al. revealed a significant change in the varus/valgus tilt between short- and long-stem femoral components 2 years after THA [22]. Computer-assisted radiographic analysis [7] exhibited neutrally aligned, short, cementless femoral stems in 56% of cases, a varus-valgus alignment of less than 5° in 36%, and an alignment of 5° or more in 8%. Hossain et al. [21] found positioning was significantly more varus in the short stem group than in the conventional stem group. Furthermore, Panisello et al. [23] found that stress transfer moved distally if stems were placed with over 5° of varus. In our study, a more than 1.5-year follow-up showed that 61% of hips had neutral alignment (0–2°), 32% had varus-valgus alignments of less than 5°, and 9% had varus-valgus alignments of 5° or more. The result suggested that thigh pain might be a sign of stem malalignment.

We evaluated the S-ICDR between the proximal end of the tip arc and the distal end of the porous coating to study the stem position relative to the adjacent femoral cortical bone. S-ICDR did not differ between these two groups. We also compared these two groups in terms of VCSA and FSS and found that they were significantly higher in the thigh pain group (*p* = 0.000 and *p* = 0.004, respectively) (Table 3). Moreover, our data were in line with the findings of other studies [24, 25]. Although the VCSA and FSS were greater in patients with thigh pain than in those without, the clinical relevance remained unclear. However, patients with unstable femoral stem fixation might experience postoperative thigh pain and more micromotions took place at the bone-implant interface, which were believed to elicit fibrous tissue formation rather than bony osseointegration [26, 27]. Banerjee et al. believed that, compared to longer uncemented components, improved proximal bone loading using a shortened stem might come at the cost of reduced primary stability, which could lead to implant migration and thus increase the risk of implant loosening and thigh pain by compromising osteointegration [28–30]. On the basis of our findings, we also believe that the use of short tapered stems reduces implant stability, increases interface micromotion, and causes thigh pain. Type I fit may be less stable and result in potting of the stem distally and distal loading, which could also contribute to thigh pain.

**Table 3:** Radiographic parameters between the pain group and the no-pain group

Variable	Thigh pain group	No thigh pain group	*p* value
Preoperative parameters			
FFI (a/b)	3.38	3.32	.525
a	3.95	4.00	.575
b	1.21	1.25	.286
FCI ((c − d)/c)	0.51	0.52	.412
c	2.53	2.61	.111
d	1.22	1.25	.497
Postoperative parameters			
S-ICDR (e/f)	0.80	0.82	.148
e	1.08	1.15	.091
f	1.39	1.41	.926
S-ICDR (g/h)	0.84	0.82	.069
g	1.76	1.80	.306
h	2.11	2.20	.088
CSA (°)	2.52	1.65	.001
SSA (°)	4.63	3.96	.016
FSS (cm)	0.29	0.12	.000
VCSA (°)	1.32	0.85	.004

*FFI* femoral flare index, *FCI* femoral cortical index, *S-ICDR* stem-intramedullary canal diameter ratio, *CSA* coronal stem angulation, *SSA* sagittal stem angulation, *FSS* femoral stem subsidence from the first to last follow-up visits, *VCSA* variation in coronal stem angulation from the first to last follow-up visits

In fact, the biomechanical and pathological mechanisms of postoperative thigh pain remain unclear. Khanuja et al. [31] reported that patients receiving short-stem replacement had a higher rate of revision surgery because of non-physiological stress transfer. In addition, cortical hypertrophy around an implant is indicative of increased stress and high-level load transfer. The impact of femoral stress shielding should be investigated further. Some researchers believe that cortical hypertrophy is associated with thigh pain and local micromotion [16, 32, 33]. However, Crawford et al. found that distal femoral cortical hypertrophy after THA using short stems was not related to thigh pain [20]. Thalmann et al. failed to find any relationship between distal, femoral cortical hypertrophy, and thigh pain [34]. More in-depth studies are warranted to fully understand the relationship among them.

In summary, a more varus/valgus stem alignment, a suboptimal stem fixation, and a higher proportion of type I fits were associated with thigh pain. We suggest that the type I fit, featuring distal contact between the stem tip and the medial femoral cortex, to some extent, is indicative of the malalignment of the implant, which, in turn, compromises implant stability, increases regional stress, and causes thigh pain.

This study has several limitations. First, this is a case series where three surgeons performed the surgery with different operative approaches, and outcomes (such as the thigh pain) might vary with different surgeons and operator bias might result. Second, although patients were asked specifically if they had “thigh pain,” it was difficult for some subjects to differentiate hip pain, lumbar spine radicular pain, pain resulting from trochanteric bursitis, and abductor tendonitis, especially when the survey was conducted over the phone. Despite all the efforts made to rule out non-implant-related causes, thigh pain could be caused by numerous causes such as undetectable neurological pathology or muscle strain. These might result in an overestimation of thigh pain. Third, the study especially lasted for a relatively short time, especially for a THA follow-up, and thigh pain may modulate over time. Forth, we focused on only one specific type of stem, and the conclusion should be extrapolated to other stems with caution. Finally, this study has similar limitations as all other radiographic studies of THA, i.e., having inter- and intra-observer variability of radiographic measurements.

## Conclusion

Our clinical and radiological analyses showed that short tapered stems could attain evident functional improvement in terms of HSS. However, stem malalignment and the distal contact between the stem tip and the medial femoral cortex might cause thigh pain. It is essential that distal implant contact be avoided and stem alignment be meticulously executed during surgical procedure. Future studies with longer follow-up and larger cohorts will provide more valuable information.

## Data Availability

This study does not contain any third material.

## Abbreviations

THA: Total hip arthroplasty
ML: Mediolateral
HHS: Harris Hip Score
AP: Anteroposterior
FCI: Femoral cortical index
FFI: Femoral flare index
CSA: Coronal stem angulation
S-ICDR: Stem-intramedullary canal diameter ratio
FSS: Femoral stem subsidence
VCSA: Variation in coronal stem angulation
SSA: Sagittal stem angulation
